RETRACTED

# Wavelet-Based Multiscale Decomposition Algorithm for Trajectory Capture of Tennis Serves

**DOI:** 10.1155/2022/3032771

**Published:** 2022-08-09

**Authors:** Shiguang Wang, Yaozhen Cui

**Affiliations:** ^1^Department of Physical Education, Yulin University, Yulin 719000, China; ^2^Department of Physical Education, Qingdao City University, Qingdao 266000, China

## Abstract

Tennis is a sport that is enjoyed by young and old alike. Participants can decide the style of play and control the speed and spin of the ball according to their ability, so the physical demands on participants are not high and the amount of exercise can be effectively controlled. With the increasing demand for quality of life, the population of tennis is growing rapidly. People have taken up tennis as a form of recreation. For professional players, the serve, as the foundation of the introduction to tennis, has been a challenge. A good serve can effectively control the situation on the court and even turn defeat into victory. Therefore, this paper focuses on capturing tennis trajectories using multidimensional wavelet segmentation in an attempt to provide an effective reference for tennis. The results show that our method has a good trajectory capturing effect and can correct and guide the tennis serving action well.

## 1. Introduction

Tennis skills include serve, forehand, backhand, net technique, and cutting and every match starts with a serve. An aggressive and successful serve will lay the foundation for the use of other skills and reduce the risk of using other skills to win the match. The evaluation of serving ability includes the success rate of the first serve, second serve, and winning percentage, which are the overall competitiveness of a good professional athlete. In a match that takes an average of 2–4 hours, the serve is the start of each point and plays a crucial role in the overall match [1].

The serve is made through the leg stirrups, then the ground reaction force on the leg, from the leg through the torso to the shoulder to the arm to the fingers, and finally to the racket, which then hits the ball. And, this process is a whipping action, from the larger joints to the small joints, although the movement of the large joints is not very fast but due to the role of the whipping, from the large joints to the small joints, so that the small joints can have rapid movement and thus act on the ball [2]. The joints that need to act in this process are: the knee, hip, thoracic spine, shoulder, elbow, and wrist joints, and the flexibility of the activities of these joints depends on their rotation, and there are major muscles and ligaments distributed around these joints [3]. A player with a strong serve should have good flexibility and stability in his serve power chain. The flexibility and stability of the knee, hip, thoracic spine, shoulder, elbow, and wrist joints are important to the serve, while the torso, as the middle link between the top and the bottom, its mobility directly affects the transfer and conversion of kinetic energy and thus directly affects the quality of the serve [4]. Even if the knee, elbow, and wrist joints are within a reasonable range, the torso cannot hit the ball at a reasonable point in time due to the unreasonable movement angle of the torso, thus affecting the serve effect.

RETRACTED

In this paper, we propose a tennis trajectory extraction method based on a multidimensional wavelet segmentation algorithm and extract the tennis trajectory under a 3D visual model. Finally, based on the experimental analysis, the advantages of the method in improving the trajectory acquisition and motion correction methods are verified. Our method has a good grip effect and can well correct and guide the tennis ball serving action.

## 2. Related Work

In “technical kinematic analysis of the serve action of outstanding reserve male tennis players in Jiangsu Province” was to record the serve action of each test player using a high-speed camera with a frequency of 300 frames/second and an exposure time of 1/2000 and then to analyze the recorded data systematically with video analysis equipment [5]. The analysis process requires the analysis of 19 points. There are 16 joints on the player's body, 2 on the racket, and 1 on the ball, and each point is processed for systematic analysis. The action analysis is performed from the preparation movement to the end of the stroke, with an average of 500 images per person [6].

In “Analysis of kinematic indexes of vigorous serving techniques of national tennis team players” two 200 Hz high-speed cameras were used to capture the player's serving movements, one machine was placed at an angle of 10–20° to the front of the player, and the other at the same angle to the front and back, with an angle of about 90° between them [7]. Have the right-handed player stand in zone one to serve first serves and the left-handed player stand in zone two to serve first serves. Before serving, tell them how the game was served and how to serve now. Each person will serve eight times each time, and the coach of each player will evaluate and record three good shots and then use the video analysis system to analyze the data. Ali, Rahman, Sungyoung Lee, and Tae Choong Chung [8] used video footage in the analysis of Djokovic's serve mechanics and tactics for each of his serves.

The biomechanical study of the effect of tennis training on the tennis serve by [9] used a high-speed video camera to film the serving action and used myoelectricity to measure the maximum force distance and the time reached at the shoulder joint in an intervention training with an elastic band to compare the differences before and after training. In the study of [10], the effect of prolonged tennis matches on the internal range of motion of the shoulder joint was studied in which passive medial and lateral shoulder rotations were calculated for 8 male tennis players every 30 minutes after 3 hours of play. All combinations of lateral and medial shoulder rotation will be calculated and ball speed will be recorded during and after the match by a radar gun. The kinetic energy transfer during the tennis serve is studied by applying two synchronized cameras recorded at 125 Hz and then analyzed using 3D photogrammetry to create five rigid bodies using 28 points on the body. High-speed cameras with different frequencies and exposures were used to record the motion of each joint in the technical tennis action, and the motion analysis system was used to analyze the recorded motion.

RETRACTED

In Palanisamy and Thangaraju et al. [11], a PTI 3D motion capture system was used to capture each player's serving motion at an interval rate of 10 m/s and 100 frames per second in a kinematic study of upper limb chain whipping action in tennis. Four capture systems were set up in four directions, with two cameras 5 m apart, and the camera with the radio receiver was set up as the main camera. Thirty-six points were selected, and 33 points were selected on the arm and torso of the racket. In addition, the racket was chosen with the sweet spot as the origin, a point at the top of the racket, and a point at the edge of the racket, and the three points were connected at right angles and labeled with marker points. Let the athletes be in the designated area, and the experimenter collects their movement data and analyzes their data one by one.

In Alsubari and Deshmukh et al. (2022) [12], the biomechanical study of four serving motions of high-level tennis players in China used the motion capture system and tachymeter to record the test data with a frequency of 120 Hz, shared 12 cameras of the same system, placed the cameras on the top of the laboratory room, and then debugged to reach the data that could record all the points of luminescence of the testers. After using the software developed to record the data of the luminous balls, a three-dimensional model of the human body is established and the data of each luminous ball are obtained, and finally, a multimedia report with charts, three-dimensional images, videos, and other information is output in the multimedia integration software.

RETRACTED

In Li and Huang (2020) [15], six cameras of the Swedish Qualisys motion capture system were used to record and analyze the ball throwing process of tennis balls, etc. The motion data of the left and right hands of the athletes were obtained, and the joint moments of the left and right hands were calculated by using the establishment of multiple rigid bodies, and the relevant formulas and methods were applied to calculate the reaction forces between the left and right hands and the momentum moments of each joint link of the left and right hands, and the dynamics of the action of each link of the upper limbs of the whipping action were analyzed. In [16], the motion capture video apparatus was applied to test and record the serving movements of tennis players, and then the kinematic and kinetic data of each player's serving movements were obtained and analyzed with related software. In 2015 [17], a Swedish infrared motion capture system was used to investigate the difference between the forehand head speed of tennis players of different levels on the accuracy of the serve and its influence.

The ITN serve test method is to divide the serve into the inner corner area and outer corner area, a total of four areas, each area serves three balls, and each ball can have two serving opportunities, a total of 12 balls [16–18].

## 3. Method

The multiscale wavelet decomposition time-frequency analysis method, also known as wavelet transform, requires the following function *φ*_*ab*_(*t*)=1/.*b*(*b* ∈ *R*) conditions to be satisfied.

(1) $$\begin{array}{c} \int_{ax}^{x}{\left|\hat{\varphi }\left(\omega \right)\right|}^{2}{\left|\omega \right|}^{-1}d\omega \;<+\infty , \end{array}$$

where the wavelet mother function is denoted as *φ*(*t*), the dependent scale factor generated from it is denoted as *a*(*a* > 0), *b*(*b* ∈ *R*) denotes the translation parameter, and the continuous wavelet of the two is denoted as follows:

(2) $$\begin{array}{c} \varphi_{ab}=\frac{1}{\sqrt{a}}\varphi \left(\frac{t-b}{a}\right). \end{array}$$

Therefore, let the signal be *f*(*t*) ∈ *L*^2^(−*∞*, +*∞*) , and convert the wavelet into the following equation:

(3) $$\begin{array}{c} aP+by+cz+d=0L3=L1\times L2,i,j,k.xy,\\ z+D=0. \end{array}$$

The wavelet transform uses the *f*(*t*) signal and *φ*(*t*) different time shifts and scale shifts for comparison and then calculates its frequency components to decompose the signal. The wavelet discretization transform is to discretize *a* and *b*. The most effective method of wavelet discretization is the Mara algorithm. It is mainly used to change the scale factor to decompose layer by layer, and each layer is decomposed to obtain the detailed part and the approximate part. Wavelet decomposition aggregates its approximation amount to blur the load transient wave signal, while the multiscale decomposition blurring varies in degree.

RETRACTED

In this paper, the feature parameters of tennis serves are extracted by mapping n-dimensional features to *k*-dimensions,and *n* > *k*. In this paper, *n*  = 8 and *k*  = 6. This*k*-dimensional variables are uncorrelated with each other and reflect enough information of the original data. Assuming a data set on the data space,

(4) $$\begin{array}{c} X={\left(x_{ij}\right)}_{n\times m}, \end{array}$$

where *x*_*ij*_ is the evaluation value of the *j* th player for some evaluation index *i*; *n*  = 1, 2, ..., 8; *m*  = 1, 2, ..., 150.

First, the raw tennis serve data are normalized by the following equation:

(5) $$\begin{array}{c} z_{ij}=\frac{\left(x_{ij}-\overset{¯}{x_{i}}\right)}{S_{i}}\;. \end{array}$$

According to experiments, the 8-dimensional vector ensures the accuracy of the data and improves the accuracy of the classification, so the 150 new 8-dimensional variables *z*_1_, *z*_2_, ..., *z*_*k*_, *k*=150, are expressed as a linear combination of *X*=(*x*_*ij*_)_*n*×*m*_ , such that the variance of the transformed new variables is minimized by the following equation:

(6) $$\begin{array}{c} \;\left\{\begin{array}{c} z_{1}=\alpha_{11}x_{11}+\alpha_{12}x_{12}+\cdots +\alpha_{1n}x_{1n}\\ z_{2}=\alpha_{21}x_{21}+\alpha_{22}x_{22}+\cdots +\alpha_{2n}x_{2n}\\ z_{3}=\alpha_{31}x_{31}+\alpha_{32}x_{32}+\cdots +\alpha_{3n}x_{3n}\\ \vdots \\ z_{k}=\alpha_{k1}x_{k1}+\alpha_{k2}x_{k2}+\cdots +\alpha_{kn}x_{kn} \end{array}\right., \end{array}$$

where *k* is the eigenvector of the covariance matrix **D** to find the eigenvalues *λ*_*i*_ and the covariance matrix **D** is

(7) $$\begin{array}{c} D=\left\{\begin{array}{cc} \mathrm{cov}\left(x_{11},x_{11}\right) & \mathrm{cov}\left(x_{11},x_{12}\right)\;\cdots \;\mathrm{cov}\left(x_{11},x_{1n}\right)\\ \mathrm{cov}\left(x_{21},x_{21}\right) & \mathrm{cov}\left(x_{21},x_{22}\right)\;\cdots \;\mathrm{cov}\left(x_{21},x_{2n}\right)\\ \vdots & \vdots \;\;\;\;\;\cdots \;\vdots \\ \mathrm{cov}\left(x_{k1},x_{k1}\right) & \mathrm{cov}\left(x_{k1},x_{k2}\right)\;\cdots \;\mathrm{cov}\left(x_{kn},x_{kn}\right). \end{array}\right.. \end{array}$$

The contribution of principal components is calculated by picking the eigenvalues *λ*_1_, *λ*_1_, ..., *λ*_*m*_ from high to low. The principal component *z*_*i*_ contribution ratio is

(8) $$\begin{array}{c} \alpha_{k}=\frac{\lambda_{i}}{\sum_{k=1}^{p}\lambda_{k}},i=1,2,\cdots ,p. \end{array}$$

In this paper, a multidimensional wavelet segmentation algorithm is proposed to extract the tennis trajectories under the 3D visual model, and a cumulative contribution rate of 85%–95% is used to reflect most of the data information and reduce the original data dimensionality. By constructing a quadratic loss function based on the structure minimization principle and replacing the inequality constraint with an equation constraint, the original problem is transformed into a problem of solving linear equations.

RETRACTED

Define the training tennis serve data sample set as: *S*={(*x*_*k*_, *y*_*k*_), *k*=1,2, ..., *N*}, where *x*_*k*_ is the input tennis serve sample, *y*_*k*_ is the output tennis serve sample, and the objective function is

(9) $$\begin{array}{c} \min\left[\frac{1}{2}\left({\left\|\omega \right\|}^{2}+\mu |\sum_{i=1}^{n}e_{i}^{2}\right)\right]. \end{array}$$

The constraint condition is

(10) $$\begin{array}{c} y_{k}=\varphi \left(x_{k}\right)\cdot w+b_{k}+e_{k}. \end{array}$$

where *e*_*k*_ is the error variable; *w* is the weight coefficient; *b*_*k*_ is the amount of deviation; and *μ* is the canonical parameter.

Introducing the Lagrangian factor *α*_*k*_, the linear system is obtained according to the KKT condition and Mercer's theorem, and the linear system is solved by least squares, and the model is expressed as follows:

(11) $$\begin{array}{c} f\left(x\right)=\sum_{k=1}^{n}\alpha_{k}K\left(x_{k},x\right)+b, \end{array}$$

where *x* is the support vector and *σ*^2^ is the kernel function parameter.

The selection of the parameter combination (*C*, *σ*^2^), the canonical parameter *C*, and the kernel function parameter *σ*^2^ need to be optimized, and the parameters in the model are optimized algorithmically to improve the prediction ability and stability of the model.

Since there are many factors affecting tennis serve, it is a high-dimensional and nonlinear model, and it is difficult to accurately reflect the tennis serve condition by using a single prediction method. Therefore, this paper proposes a tennis serve normality prediction method based on improved PPL. The flow chart of the tennis serve normality prediction model is shown in Figure 1. For the existence of strong coupling nonlinear relationships among many influencing factors of tennis serve, the selected feature vectors are first subjected to principal component analysis, and the relevant multifactor indicators are extracted and combined into a few uncorrelated composite indicators to reduce the influence of tennis serve data correlation on the model. The extraction results were input into LSSVM and optimized by the PSO algorithm to build a tennis serve normality prediction model with higher fitting accuracy and generalization performance.

RETRACTED

The feature point distribution of tennis serve trajectory linear local information, to realize the image acquisition, and get the acquisition model as shown in Figure 2.

Through the above-given analysis, the algorithm is used to adjust and correct the captured trajectory lines to achieve the correct capture of trajectory lines, and the implementation flow of the algorithm is shown in Figure 3.

## 4. Experiments

This study focuses on the shoulder and hip kinematics in the serving action of tennis players from a sports university. There are 16 male and female athletes in a sports university tennis team, among which 7 female athletes and 9 male athletes are from the College of Athletic Sports. Among them, 5 male athletes used both FB technique and FU technique, and all 7 female athletes used the FB technique. (FU technique is the serve-up technique and FB technique is the serve-no-step technique) See Table 1.

These two measurements are that the first one was carried out during the summer vacation. At that time, the school team only had students who promised to participate in the competition, so the number of students was very small. The new members of the school team measured at the beginning of September of the academic year.

This experiment used Qualisys infrared camera (six lenses) to film the athletes' serving action. The lighted ball was placed on the neck, shoulder peaks, left and right anterior superior iliac spine, waist, and handle of the athlete, and the experimental apparatus was placed before the experiment, and the experimental apparatus was placed as shown in Figures 4 and 5.

Subjects wore tight-fitting short sleeves and shorts and finished serving in the designated area. That is, serve from zone one to zone two and each corner to serve 3 balls, each ball has two opportunities to serve. If the first serve enters the designated target area, 4 points will be awarded; otherwise, 0 points will be awarded, and if it only enters the target area, 2 points will be awarded; if the first serve misses, the second serve will be awarded, 2 points will be awarded; otherwise, 0 points will be awarded, and if it only enters the target area, 1 point will be awarded. After a valid hit, if the second bounce is not within the strength zone, no additional points are added; if the second bounce lands within the strength plus zone, such as a bonus zone (between the baseline and the double plus zone), the final score of this ball is added one point to the corresponding score of the first landing point, such as in the double score zone (4.57 m from the ends of the baseline and 4.87 m from the midpoint of the baseline), the final score is twice the score of the first point. The calculation of the basic axis and the basic section of the human body is as follows.

RETRACTED

The coordinates corresponding to the basic axes and basic sections of the human body can be calculated from the image screen analysis. The following equation shows the horizontal, vertical, and vertical coordinates of each body measurement point.

Human frontal axis: (1) right shoulder ⟶ left shoulder (calculate upper limb joint angle), or right hip ⟶ left hip (calculate lower limb joint angle) *L*1 = (right shoulder horizontal coordinate - left shoulder horizontal coordinate) *i* + *j* + *k* or *L*1 = (right hip horizontal coordinate - left hip horizontal coordinate) *i* + (right hip vertical coordinate - left hip vertical coordinate) *j* + (right hip vertical coordinates - left hip vertical coordinates) *k*.

(2) Human body vertical axis: neck point ⟶ umbilical point (or the midpoint of the two shoulder line ⟶ the midpoint of the two hip lines), *L*2 = (umbilical horizontal coordinates - neck horizontal coordinates) *i* + (umbilical vertical coordinates - neck vertical coordinates) *j* + (umbilical vertical coordinates - neck vertical coordinates) *k*.

The sagittal axis of the human body is the vector product of the frontal of the human body *L*3=*L*1 × *L*2. From the body basic axis can determine the plane equation of the body basic tangent plane.

Body horizontal plane: the plane with the body vertical axis as the normal vector.

(umbilical horizontal coordinate - neck horizontal coordinate) *x* + (umbilical vertical coordinate - neck vertical coordinate) *y* + (umbilical vertical coordinate - neck vertical coordinate) *z*+*D*=0

(3) (right shoulder transverse coordinate) *x* + (longitudinal coordinate) *y* + (vertical coordinate) *z*+*D*=0 or (right hip transverse coordinate - left hip transverse coordinate) *x* + (right hip longitudinal coordinate - left hip longitudinal coordinate) *y* + (right hip vertical coordinate - left hip vertical coordinate) *z*+*D*=0.

The frontal plane of the human body: *ax*+*by*+*cz*+*d*=0. In the above equations, *D* is the coefficient to determine the plane position and its exact value is not necessary to know in the later calculation.

(4) In addition, when calculating the upper arm rotation, forearm rotation, and wrist angle, the plane normal to the long axis of a link is also calculated according to the specific situation. For example, the plane perpendicular to the upper arm: (elbow transverse coordinate - shoulder transverse coordinate) *x* + (elbow longitudinal coordinate - shoulder longitudinal coordinate) *y* + (elbow longitudinal coordinate - shoulder longitudinal coordinate) *z*+*D*=0. The plane perpendicular to the forearm: (wrist transverse coordinate - elbow transverse coordinate) *x* + (longitudinal coordinate wrist - elbow longitudinal coordinate) *y* + (wrist vertical coordinate - elbow vertical coordinate) *z*+*D*=0.

RETRACTED

See Figure 6 for double plus line diagram, Figure 7 for player front lighted ball placement, Figure 8 for player back lighted ball placement, and Figure 9 for the serve target area and designated target area.

In this study, the independent sample *t*-test was conducted and the independent sample *t*-test of the shoulder-hip torsion angles of male and female athletes at the moment of tossing and racket lifting in the first shot. The independent sample *t*-test of the second serve toss was found; the independent sample *t*-test of the second serve for both male and female athletes was found that there was no significant difference between them *P*  = 0.382 (*P* > 0.05). It shows that the shoulder and hip torsion angles of girls and boys at the moment of raising the racket and at the moment of hitting the ball in the first and second serves is not different. The division of girls' serving score steps is shown in Table 2.

See Table 3 for the breakdown of the men's serving score ladder.

In this paper, the ITN serve test scores are used to distinguish the serve levels. According to the division of ITN level table is divided into a total of 10 segments, the total ITN test score is 430 points, the total serve score is 108 points, the ratio of these two is approximated by 0.25, that is, the serve score of boys ITN1 (363–430 points) is 91–108 points, the serve score range of girls ITN1 (345–430 points) is 86–108, if the serve is within the range of ITN1 The boys' ITN2 (338–362) serve score range is 84–90 and the girls' ITN2 (304–344) serve score range is 76–85, if the serve score is within the ITN2 range is classified as the second step; the boys' ITN3 (294–337) serve score is 73–83 and the girls' ITN3 (259–303) were scored 65–75 if the serve score was in the ITN3 range and were classified as the third order; boys ITN4 (269–293) were scored 67–72 if the serve score was in the ITN4 range and girls ITN4 (231–258) were scored 58–64 if the serve score was in the ITN4 range and were classified as the fourth order. The serving scores of male and female athletes in this study were divided into steps, and the serving shoulder and hip trajectories of male and female athletes in the horizontal plane were compared to find out the differences between them. The following analyzes were performed.

We can find the serve trajectory as in Figure 10 in the horizontal plane of the shoulder-hip movement up and down obviously, reaching the highest point at the time of hitting the ball.

RETRACTED

For boys, according to their serve shoulder-hip activity in the horizontal plane of the up and down undulation trajectory is shown in Figure 11, the shoulder-hip relative rise height ratio of the second step male athletes is shown in Table 4.

To capture and extract features of tennis serve trajectories, simulation experiments were conducted in Matlab. The line capture frequency was 16 kHz, and the line capture function such as received in Matlab was invoked to capture the lines of the tennis ball trajectory. Firstly, the computer 3D visual acquisition of tennis trajectory was carried out, and the original image acquisition and filter image was shown in Figures 12 and 13.

Based on the feature extraction results in Figure 13, we implemented the trajectory line capture of the tennis serve and tested the accuracy of different trajectory capture methods. The comparison results are shown in Figure 14. The computational overheads of different methods are depicted in Table 5.

Analysis of the above-given results shows that the performance of our method is high and the computational overhead is low.

## 5. Conclusion

The accuracy of tennis service can be improved by capturing the trajectory of tennis serving, trajectory analysis, and image processing technology. In this paper, we propose a comprehensive method to capture tennis trajectory in a three-dimensional visual model. In general, this paper effectively extracts the tennis service trajectory and extracts the edge information of the service trajectory through the method of wavelet analysis, which can not only correct the service action but also repeat the service action and self-examination of the players, which is undoubtedly very valuable for tennis. The experimental results also show that our method not only has high capture accuracy but also has good real-time performance, and can well adapt to the real-time capture of tennis trajectory.

## Figures and Tables

**Figure 1:** Flow chart of tennis serve normality model.

**Figure 2:** Image acquisition model of tennis serve trajectory.

**Figure 3:** Flowchart of algorithm implementation.

**Figure 4:** Serving partition.

**Figure 5:** Apparatus placement.

**Figure 6:** Double plus line graph.

**Figure 7:** Athlete front lighted ball placement diagram.

**Figure 8:** Athletes back-lit ball placement.

**Figure 9:** Serve target area, designated target area.

**Figure 10:** Trajectory of the up and down of the girls' serve shoulder and hip activity in the horizontal plane.

**Figure 11:** Trajectory of up and down of shoulder and hip activities in horizontal plane for boys serving.

RETRACTED

**Figure 12:** Original image acquisition.

**Figure 13:** Feature extraction results.

**Figure 14:** Comparison of accuracy of trajectory capture.

**Table 1:** Basic information of male and female athletes.

Gender	Age (years)	Height (cm)	Weight (kg)	FB technology	FU technique
Male athletes	19.65 ± 1.062	183 ± 4.528	71.77 ± 5.652	5	5
Female athletes	20.01 ± 2.01	170.85 ± 3.192	59.34 ± 3.725	0	7

**Table 2:** Girls' serving score ladder.

Ladder division	Shoulder hip twist angle when raising the racket in one shot	Shoulder hip twist angle at first shot	The angle of shoulder-hip twist when raising the racket for the second shot	Shoulder hip twist angle during the second shot
First level ladder	28.315	39.531	28.82	37.25
Secondary ladder	28.645	35.272	39.0968	40.534
Third step	31.517	44.257	28.116	43.766
Fourth step	32.797	36.178	33.954	47.238

**Table 3:** Men's serving score ladder division.

Ladder division	Shoulder hip twist angle when raising the racket in one shot	Shoulder hip twist angle at first shot	The angle of shoulder-hip twist when raising the racket for the second shot	Shoulder hip twist angle during the second shot
Secondary ladder	33.847	35.678	30.4039	41.579
Third step	35.193	29.457	33.444	30.847
Fourth step	21.124	26.729	28.1025	36.159

**Table 4:** Relative rise height ratio of male athletes in the second step ladder.

First and second shot shoulder and hip strike relative rise height ratio	Wu ×	Chen ×	Liu ×	Bai ×	Average relative altitude rise ratio
First shot shoulder and hip strike relative rise height ratio	0.057	0.066	0.065	0.066	0.0632
Second shot shoulder and hip strike relative rise height ratio	0.07	0.065	0.062	0.067	0.06281

**Table 5:** Comparison of computational overhead/s.

# Iterations	Our method	Literature [3]	Literature [4]
100	0.11	0.47	1.44
200	0.06	0.88	1.87
300	0.07	1.25	2.01

## Data Availability

The experimental data used to support the findings of this study are available from the corresponding author upon request.
